The article "Mesenchymal stem cells in the osteosarcoma microenvironment: their biological properties, influence on tumor growth, and therapeutic implications" was published in 2018. Journal: Stem Cell Res Ther.

# Mesenchymal stem cells in the osteosarcoma microenvironment: their biological properties, influence on tumor growth, and therapeutic implications

**DOI:** 10.1186/s13287-018-0780-x

**Published:** 2018-01-31

**Authors:** Ying Zheng, Gangyang Wang, Ruiling Chen, Yingqi Hua, Zhengdong Cai

**Affiliations:** Department of Orthopaedics, Shanghai Bone Tumor Institute, Shanghai General Hospital, Shanghai Jiao Tong University School of Medicine, 100 Haining Road Shanghai, Shanghai, China

**Keywords:** MSCs, Osteosarcoma, Metastasis, Drug resistance, Clinical applications

## Abstract

During tumorigenesis and development, participation of the tumor microenvironment is not negligible. As an important component in the tumor microenvironment, mesenchymal stem cells (MSCs) have been corroborated to mediate proliferation, metastasis, and drug resistance in many cancers, including osteosarcoma. What’s more, because of tumor site tropism, MSCs can be engineered to be loaded with therapeutic agents so that drugs can be precisely delivered to tumor lesions. In this review, we mainly discuss recent advances concerning the functions of MSCs in osteosarcoma and their possible clinical applications in the future.

## Background

Osteosarcoma (OS) is a malignant bone tumor and usually afflicts people in adolescence. Nowadays, neoadjuvant chemotherapy combined with conservative surgical resection and post-operative adjuvant chemotherapy is the preferential treatment for OS patients. However, because of distant metastasis and chemotherapy resistance, efficacy is still unsatisfactory. Local tumor microenvironments (TMEs) comprise extracellular matrix and cellular components [1] and, over the years, the TME has been documented to be firmly associated with the initiation and progression of OS and to contribute its poor prognosis. In the TME, non-tumor cells such as fibroblasts, endothelial cells, immune cells, and MSCs play important roles in tumor development [2]. Notably, a growing body of evidence has implied the involvement of MSCs in OS progression.

MSCs are non-hematopoietic precursor cells and have been found in many human tissues, such as bone marrow, adipose tissue, peripheral blood, placenta, and umbilical cord [3, 4]. They also exhibit an ability to self-renew and differentiate into a variety of mesenchymal cell lineages, like osteocytes, chondrocytes, and adipocytes [5].

Recently, MSCs have been considered to participate in wound healing [6, 7]. As “wounds that never heal”, tumors are also conjectured to be influenced by MSCs. Prior reports have provided results that although they share similar characteristics with regard to morphology and multilineage differentiation capability, MSCs from tumor tissue (T-MSCs) and MSCs from normal tissue (N-MSCs) have different impacts on tumor development [8]. For instance, in Ewing sarcoma, T-MSCs exhibit a significantly greater proliferative capacity than N-MSCs [9]. Under the influence of tumor cells and chronic TME, circling N-MSCs migrate to tumor lesions and are “educated” to be T-MSCs that support the growth of tumor. Moreover, after MSCs are recruited to the tumor lesions, they can obtain a specific tumor-associated fibroblast (TAF) phenotype and encourage tumor cell growth [10]. A large amount of cytokines secreted by the TME and tumor cells are involved in this process, including interleukin (IL)-6, transforming growth factor (TGF)-β, stromal-derived factor (SDF)-1, tumor necrosis factor (TNF)-α, interferon (IFN)-γ, macrophage inhibition factor (MIF), and IL-1α [8, 11] (Fig. 1). In this review, we discuss the role of MSCs in OS and their potential treatment applications based on the findings from recent studies.

The article "Mesenchymal stem cells in the osteosarcoma microenvironment: their biological properties, influence on tumor growth, and therapeutic implications" was published in 2018. Journal: Stem Cell Res Ther.

**Fig. 1:** Different effects exerted by the TME on naïve MSCs (*N-MSC*). Under the effects of some cytokines (SDF-1, MIF, TGF-β, and so on), N-MSCs are recruited to the TME. Through the paracrine network in the TME, N-MSCs undergo a series of functional transformations. On one hand, INF-γ, TNF-α, and IL-1α strengthen the tumor growth-promoting effects of MSCs; On the other hand, INF-γ, TNF-α, and TGF-β enhance the ability of MSCs to promote tumor metastasis. Furthermore, MSCs can differentiate into cancer-associated fibroblasts (*CAF*) under the stimulation of TGF-β

## MSCs and the biogenesis of OS

OS is characterized by a variety of histopathologic subtypes, suggesting the hypothesis that MSCs may be the origin of OS cells. According to previous investigations, mutation of related genes [12], the differentiation stage of MSCs [13], the tissue source of MSCs [13], and the bone environment [14] can influence the malignant transformation of MSCs.

In vivo research found that the overexpression of c-MYC with loss of Ink4a/Arf could induce the malignant transformation from bone marrow-derived MSCs (BM-MSCs) to OS [15]. Wang et al. conducted research to evaluate the impact of mutation of c-MYC, Ras, Rb, and P53 on the transformation of MSCs [12]. The results demonstrated that Rb silencing and c-MYC overexpression in MSCs were associated with OS tumorigenesis [12]. Under other oncogenic stresses, however, BM-MSCs expressing the FUS-CHOP fusion gene were reported to develop as liposarcoma [16]. As such, the mesenchymal tumor histological type may be firmly linked with the type of oncogenic stress.

Except for undifferentiated MSCs, osteogenic lineage-committed progenitor cells can also become the origin for OS. It was documented that undifferentiated p53^−/−^ and Rb^−/−^ p53^−/−^ BM-MSCs led to the generation of leiomyosarcoma in vivo [13]. Interestingly, after BM-MSCs differentiated to the osteogenic lineage and were treated with p53 and Rb genes excised, they developed into tumors displaying clear OS histological features [13]. Moreover, when researchers prolonged the time of differentiation toward the osteogenic lineage, the degree of OS differentiation increased as well [13]. All these findings imply that it may be much more appropriate to classify the cellular origin of OS as “a MSC population” that is generated from MSCs induced by a specific oncogenic stress in a specific differentiation stage. The researchers also reported that none of the Rb^−/−^ p53^−/−^ ASC-derived osteogenic progenitors and undifferentiated ASCs (adipose derived MSCs) developed to be OS-like tumors in vivo [13]. Accordingly, the generation of OS may also rely on the tissue source of MSCs. Of course, we cannot exclude the possibility that ASCs with other transforming mutations will develop to be OS.

The article "Mesenchymal stem cells in the osteosarcoma microenvironment: their biological properties, influence on tumor growth, and therapeutic implications" was published in 2018. Journal: Stem Cell Res Ther.

The bone environment is yet another factor affecting differentiation. In one study, the MSCs isolated from OS were described to become the progenitor cells of OS after they had been injected into nude mice [17]. In vitro, however, the MSCs could still differentiate into osteoblasts, chondrocytes, and adipocytes. Rubio et al. [14] inoculated GFP-tagged wild type, p53^−/−^, RB^−/−^, and p53^−/−^ RB^−/−^ MSCs into NSG immunodeficient mice to investigate whether bone environment would influence the transformation of MSCs. They provided evidence that only p53^−/−^ and p53^−/−^ RB^−/−^ MSCs developed into OS-like tumors in the recipients’ bone. At the same time, tumoral positions far away from the host bone exhibited a different pathology, with the tumor resembling leiomyosarcoma much more than OS [14]. These results show that the host bone environment might be another factor in programming the sarcoma phenotype of transformed MSCs. Bone morphogenetic protein (BMP)-2 and calcium substrates are abundant in the bone milieu [14]. BMP-2 was shown to affect the osteoblastic differentiation of p53^−/−^ RB^−/−^ MSCs through autocrine activation of WNT ligands [18], thereby leading to OS phenotype development. Calcium substrates can also contribute to the development of p53^−/−^ RB^−/−^ MSC osteogenesis [19]. In light of this, researchers established a ceramic bone-like environment model to analyze the impact of the calcified extracellular matrix on the osteogenesis and sarcomagenesis potential of p53^−/−^ RB^−/−^ MSCs [14]. In the absence of BMP-2, the tumor showed a small area of osteogenic differentiation that just surrounded the ceramic material; however, when BMP-2 was added to the ceramic-fibrin structure, the OS-like tumor occupied a much larger area [14]. Consequently, bone environment signals can influence the differentiation of distinct sarcoma phenotypes.

The article "Mesenchymal stem cells in the osteosarcoma microenvironment: their biological properties, influence on tumor growth, and therapeutic implications" was published in 2018. Journal: Stem Cell Res Ther.

## Promotion of OS growth

### Proliferation

Cancers require a sufficient energy supply for development. What’s more, they have to escape autologous immune surveillance that is usually initiated by NK cells and CD8^+^ T cells. Tumor cells are able to secret copious cytokines, like SDF-1, IL-6, and platelet-derived growth factor (PDGF), that can induce MSCs to migrate to tumor tissue [8]. On one hand, cross-talk between MSCs and tumor cells favors angiogenesis and finally creates a network of new vessels in tumor tissue. On the other hand, some cytokines secreted by MSCs, such as TGF-β, can blunt the antitumor immune responses and facilitate tumor immune escape [20].

Mohseny et al. [21] sorted three different types of low-passage MSCs (normal MSCs), high-passage MSCs (transformed MSCs), and tumorigenic MSCs (representative of OS-producing cells) through diverse times of passage. By analyzing whole-genome expression, they found that, in transformed and tumorigenic MSCs, expression of a T-cell response-associated gene (Fut-7) and major histocompatibility complex-related genes (H2-K1 and H2-D1) was reduced, while the pro-angiogenic gene Est1 was upregulated [21]. These results indicate that early OS is endowed with angiogenesis and immunosuppressive properties. Vascular endothelial growth factor (VEGF) is a classic cytokine that can activate the PI3K-Akt pathway and contribute to angiogenesis [22]. Some other cytokines such as IL-6 and Monocyte chemoattractant protein (MCP)-1 are also linked with the PI3K-Akt pathway [23]. The growth-promoting effect of IL-6 and VEGF secreted by MSCs has been verified in many studies when MSCs are co-cultured with OS cells [24–26]. As a form of intercellular communication, extracellular vesicles’ (EVs) effects on recipient cells are usually dependent on their cargos. In recent studies on OS-derived EVs, exosome-like EVs released by OS could be internalized by MSCs and the educated MSCs promoted the growth and metastasis of OS [27]. Follow-up studies implied the involvement of an inflammatory loop in which TGF-β in OS EVs induced the production of IL-6 in MSCs, activated the IL-6/STAT signaling axis in OS cells, and promoted the growth of OS in vivo [27]. Furthermore, OS can also inhibit the osteogenic differentiation of MSCs, strengthening the pro-tumor effects of MSCs [28].

### Metastasis and migration

Lung is the preferred metastatic target organ in OS. Via interclonal co-operation, highly metastatic clonal variants of OS can induce poorly metastatic clonal variants of the same cell line into a migratory and invasive phenotype [29]. During the process of horizontal phenotypic transfer, EVs wrapped with metastasis-associated proteins were released by highly metastatic OS clonal variants and internalized by poorly metastatic clonal variants. The results show that OS with high heterogeneity can strengthen its metastasis via unidirectional EV-mediated interclonal cooperation. The lung tropism of EVs also implies that lung is the preferred target organ for the establishment of a pre-metastatic niche [29].

The article "Mesenchymal stem cells in the osteosarcoma microenvironment: their biological properties, influence on tumor growth, and therapeutic implications" was published in 2018. Journal: Stem Cell Res Ther.

Emerging evidence has demonstrated the metastasis-promoting effects of MSCs on OS. Under the stimulation of human MSCs, pulmonary metastasis was promoted and some cytokines such as CCL5 (CC chemokine ligand5) and VEGF may be responsible for the migration [25, 30]. Another study documented that VEGF secreted by MSCs promoted the metastasis through elevating the expression of CXCR4 (CXC chemokine receptor4) in OS cells [26]. The hypoxic environment in cancer results from the rapid proliferation of tumor cells [31]. A recent investigation demonstrated that hypoxia together with some chemoattractants such as IL-6 and MCP-1 could recruit MSCs to tumor lesions. Via the cross-talk between MSCs and tumor cells, the secretions, e.g., CCL5, placenta growth factor (PIGF) and CXCL10 promoted the metastasis of malignant cells [32]. When the hypoxia persisted, the metabolic process of the cells switched to continuous anaerobic glycolysis, and subsequently induced tumor-associated extracellular acidification [32]. In another study, short-term acidification was described to convert MSCs to T-MSCs [33]. Moreover, via the activation of the NF-κB pathway, T-MSCs secreted some clonogenicity-related and migration-related factors such as CCL-5 [33]. This study demonstrated that tumoral acidosis was crucial in the migration, which was usually ignored in the past.

In the model of cancer stem cell (CSC) theory, CSCs originate from stem cells or precursor cells with epigenetic mutations. They can form and sustain tumors and are resistant to traditional therapies [34]. Many studies have provided evidence for the existence of stem-like properities in OS [35, 36]. Under the influence of MSCs, OS cells can also acquire the phenotype of stem cells [24, 33]. What’s more, CSCs can stimulate MSCs to secret TGF-β1, which induces NF-kB gene activation in MSCs and subsequent IL-6 secretion by MSCs [24]. After that, the expression of some prometastatic genes, including intercellular adhesion molecule-1 and MET, is elevated [24]. The cellular interaction based on cytokines is critically important, and some investigations also showed the importance of horizontal gene transfer among cells for tumor aggressiveness. An investigation demonstrated Ki-ras gene transfer from 143B-GFP cells (OS cells with high metastatic potential) to MNNG/HOS-RFP cells (OS cells with low metastatic potential) in vivo. The metastasis of MNNG/HOS-RFP was enhanced in response [37]. Whether gene transfer between OS cells and MSCs cells promotes OS needs to be further explored.

The article "Mesenchymal stem cells in the osteosarcoma microenvironment: their biological properties, influence on tumor growth, and therapeutic implications" was published in 2018. Journal: Stem Cell Res Ther.

### Drug resistance

MSCs can foster the stemness of tumor cells. Through the following mechanisms, CSCs can strengthen their tolerance to chemotherapeutics: first, upregulated expression of drug efflux pumps (Pgp and ABCG2); second, more active ALDH (aldehyde dehydrogenase), which has been demonstrated to confer resistance to cyclophosphamide; third, increased expression of pro-survival BCL-2 (B-cell lymphoma-2) protein family members; and last but not least, strengthened DNA damage repair [38]. Furthermore, cross-talk between tumor cells and MSCs can also protect tumor cells from lethal [39]. Many products of MSCs, such as SDF-1, contribute to the drug resistance of tumors [39].

With regard to short-term acidification, MSCs were shown to secret some pro-inflammatory factors such as IL-6 and IL-8 and fostered the stemness of HOS cells [33]. As a result, OS cell sensitivity to DXR was reduced [33]. Another study showed that MSCs promoted the survival of OS cells treated with cisplatin and DOX [40]. Subsequent investigations documented that, via the activation of STAT3, IL-6 secreted by MSCs promoted the expression of MDR-1 (Multi-drug resistance gene 1) and MRP (Multidrug resistance-associated protein), which work as a drug efflux pump [40]. Collectively, MSCs play an important role in drug resistance of OS, through increasing the expression of multi-drug resistance genes or inducing the OS cells’ stemness in a paracrine pathway.

### Inhibition of OS growth

Even though many researchers have reported that MSCs support OS growth, a few studies have also shown that MSCs suppress OS growth. Wharton’s jelly-derived MSCs (WJ-MSCs) are homogeneous populations of MSCs isolated from the gelatinous Wharton’s jelly in the umbilical cord. When OS cells (MG-63) were cultured in human WJ-MSC-conditioned medium, their growth, including proliferation and migration in vitro, was inhibited [41].

Taken together, the previous studies on the effects of MSCs on tumor development have demonstrated contradicting results. Even though the reasons for these contradictions are yet to be explored, it can be inferred that the results are affected by many aspects, including the TME, the source of MSCs, the type of tumor, the methodologies of the experiments, and the animal model. As a special type of MSC, WJ-MSCs have been reported to attenuate the growth of many tumors, including OS [41]. According to this, WJ-MSCs may be safe for future clinical applications. The details of some roles of MSCs in OS are shown in Table 1.

The article "Mesenchymal stem cells in the osteosarcoma microenvironment: their biological properties, influence on tumor growth, and therapeutic implications" was published in 2018. Journal: Stem Cell Res Ther.

**Table 1:** Some roles of MSCs in OS

Function	Source of MSCs or other related cells	Type of OS cells	Relevant molecules or genes	References
Differentiating to OS	Mouse bone marrow and adipose tissue	/	P53 knockout	[14]
		/	P53 and Rb knockout	[14]
	Mouse bone marrow	/	c-MYC overexpression and Ink4a/Arf knockout	[15]
	Osteochondrocyte progenitors	/	c-MYC overexpression and Ink4a/Arf knockout	[15]
	Human bone marrow	/	c-Myc overexpression and Rb silencing	[12]
	Mouse	/	Loss of Cdkn2a/p16	[17]
	Osteogenic lineage-committed progenitor cells	/	P53 and Rb knockout	[13]
Promoting proliferation	Bone marrow	Tumorigenic MSCs	Gene (Fut-7, H2-K1, and H2-D1)↑; Gene (Est1)↓	[21]
	Bone marrow	HOS-CSC	TGF-β-dependent IL-6 secretion	[24]
	Human	9607-F5M2	CXCR4-mediated high expression of VEGF	[26]
	Human	Saos-2	CCL5 secreted by hMSCs	[30]
	Human adipose tissue	MG63, HOS, and 143B cells	IL6 secretion induced by OS EVs	[27]
Promoting metastasis	Bone marrow	UMR-106	High expression of VEGF	[25]
	Human	9607-F5M2	CXCR4-mediated high expression of VEGF	[26]
	Human	Saos-2	CCL5 secreted by human MSCs	[30]
	Bone marrow and adipose tissue	MG-63, Saos-2, and HOS	IL6, IL8, CCL5, GM-CSF, CXCL1, and CXCL5 secreted by activated MSCs, promoting stemness	[33]
	Human adipose tissue	MG63, HOS, and 143B cells	IL-6 secretion-induced by OS EVs	[27]
Strengthening drug resistance	Bone marrow and adipose tissue	MG-63, Saos-2, and HOS	IL6, IL8, CCL5, GM-CSF, CXCL1, and CXCL5 secreted by activated MSCs, promoting stemness	[33]
	Human bone marrow	Saos-2 and U2-OS	IL-6/STAT3 signaling	[40]
Inhibiting proliferation and migration	Wharton’s jelly	MG-63	Beclin-1 and LC3B	[41]

## The prospects of MSCs in clinical applications

### Delivering agents to OS tumors

MSCs have tropism toward tumor stroma. Taking advantage of this characteristic, we can load MSCs with therapeutic agents and utilize their anti-cancer effects more effectively. In a study, murine ASCs were transfected with the full-length human TRAIL (TNF-related apoptosis-inducing ligand) gene, which has been reported to induce death in OS [42]. The experiment in vitro showed that TRAIL delivered by MSCs significantly induced the apoptosis of SAOS2 via the activation of caspase-8 [3]. After MSCs were transfected with adenoviruses that carried the osteoprotegerin gene, they were also reported to suppress the growth of OS and bone destruction [43]. Except for being transfected with some pro-apoptosis genes, MSCs can also be modified to deliver medicine. Generally speaking, the cargos MSCs carry should possess at least the following four characteristics: 1, strong toxicity towards tumor tissue; 2, non-deleterious to the MSCs during migration; 3, not affected by the MSCs; 4, not affect the biological properties of the MSCs.

The article "Mesenchymal stem cells in the osteosarcoma microenvironment: their biological properties, influence on tumor growth, and therapeutic implications" was published in 2018. Journal: Stem Cell Res Ther.

Traditional chemical drugs as cargos in MSCs would possibly ruin the MSCs, which will make the drug delivery fail. Because of this, photodynamic therapy may be a good choice. Duchi et al. [44] loaded a photosensitizer (TPPS) into core-shell PMMA nanoparticles (FNPs) and incorporated the compound into MSCs. When the human OS cell line U2OS-RFP-TUBA1B was co-cultured with MSCs that were loaded with TPPS-FNPs in vitro, the MSCs released reactive oxygen species and killed the surrounding tumor cells under the stimulation of photoactivation. In the process, the MSCs were also induced to die and the safe clearance of MSCs was ensured [44]. Apart from cytotoxic agents and viral vectors, anti-angiogenic agents and immunostimulatory agents have also been reported to be transported to tumor lesions by MSCs [45]. Promising procedures for using MSCs as delivery vehicles are shown in Fig. 2 [46, 47]. Compared with other drug carriers, such as liposomes and magnetic beads, MSCs possess particular advantages, including specific targeting, easy availability, and good immunological compatibility [45].

**Fig. 2:** Promising methods for using MSCs as delivery vehicles. (i) Transduct MSCs with retroviral vectors that carry therapeutic RNA: capture the MSCs from the patient, modify MSCs by transduction with retroviral vectors at the first passage, culture the transducted MSCs for several days, select the cells with puromycin, expand the transducted and selected cells to the clinical necessary dose, and finally administer them to the patient. (ii) Load MSCs with nanoparticles incorporated with drugs: load chemotherapeutic agents in nanoparticles, uptake the nanoparticles with MSCs, and administer the MSCs into patients

As a highly heterogeneous disease, OS usually exhibits different phenotypes in different patients. Identifying the specific phenotypes as therapeutic targets may lead to a better prognosis. Recently, researchers performed molecular profiling in two cases of OS. Even though they used sirolimus + crizotinib and abraxane + celecoxib to match the P1K3CA, c-MET, and SPARC and COX2 mutations in patient 1 and used temsirolimus, sorafenib, and bevacizumab to match NF2, PDGFRα, and TP53 mutations in patient 2, the prognosis of the two patients was still bad [48]. However, the result doesn’t mean that personalized targeted therapy is not feasible for the treatment of OS, and MSCs may exhibit their advantages in carrying targeted drugs or anti-cancer genes for personalized medicine.

The article "Mesenchymal stem cells in the osteosarcoma microenvironment: their biological properties, influence on tumor growth, and therapeutic implications" was published in 2018. Journal: Stem Cell Res Ther.

### Targeting upstream and downstream modulators of MSCs

Through the exchange of cytokines between MSCs and OS cells, cross-talk can be established to mediate the development of OS. Via targeting upstream and downstream modulators of MSCs, we can block the cross-talk and inhibit tumor progression. The SDF-1/CXCR4 axis is well-known for its pleiotropic role in tumor development [49]. Some antagonists of the CXCR4 receptor, such as AMD3100, have been developed to disturb the cross-talk [49]. Scientists employed a novel antagonist of CXCR4 named ‘Peptide R’ to inhibit BM-MSC-mediated OS [49]. The results showed that Peptide R suppressed the migration and invasiveness of U2OS through ceasing the Ras/ERK and PI3K/Akt activation that were mediated by BM-MSCs [49]. Some new medicines, such as the IDO inhibitor 1-methyl-DL-tryptophan (1-MT), can enhance the activity of antitumor T cells [50]. Even though no investigations have been carried out on the effects of IDO inhibitors on OS, strategies that reverse the immunosuppression mediated by MSCs may be promising for combination with other immunotherapies.

### Promoting bone reconstruction in OS patients

After large segment resection of tumor, OS patients are usually confronted with many challenges in the process of bone reconstruction, such as infection and local recurrence. MSCs have the ability to migrate to the wound and promote wound healing through transforming the inflammatory microenvironment [51]. With the maturity of 3D printing technique, personalized bone reconstruction supported by MSCs is developing [52]. Therefore, MSCs have potential for therapeutic use in limb salvage after tumor resection. To study their feasibility in the clinical setting, researchers inoculated mice with DLM8-luc OS cells and performed resection of the primary tumor when the OS model had developed [53]. After that, they separated the mice into three ASC treatment groups (the mice received intravenous MSCs, MSCs at the surgical area, or no MSCs). By comparing the number of pulmonary nodules, the time to first evidence of metastasis, and the size of the recurrent OS, the researchers reported that the mice that received intravenous MSCs healed much faster than the other two groups, while the development of local recurrence and the size of recurrent tumors showed no apparent difference in the three groups [53]. So it might be promising to use MSCs to augment bone healing in patients with lesions after surgery.

The article "Mesenchymal stem cells in the osteosarcoma microenvironment: their biological properties, influence on tumor growth, and therapeutic implications" was published in 2018. Journal: Stem Cell Res Ther.

Nevertheless, we have to be aware of possible relapse after the administration of MSCs. Recently, Perrot and colleagues [54] reported an unexpected late local recurrence of human OS that occurred at the site of autologous fat grafts 13 years after the initial pathology and 18 months after a lipofilling procedure. The results of their further experimental model implied the possible OS-promotion role of MSC-like cells that were contained in the fatty tissues [54]. In another study, researchers addressed that SAOS2 OS cells could maintain human ASCs in a “stemness” state which would exacerbate OS growth and aggressiveness [55]. In this manner, the remaining OS cells after resection may develop quickly under the stimulation of the MSC-like cells in the autologous fat grafts. Combined with the OS-promoting effects of MSCs we introduced above, we have to realize that the clinical applications of MSCs for OS treatment must be carefully performed after deciding on the originating tissue of MSCs, the number of MSCs, the time of MSC injection, and so on. Only when no risk of OS promotion is detected in animal experiments will MSCs meet the regulatory requirements [56].

## Conclusions and prospects

Nowadays, more and more researchers are focusing on the effects of MSCs on wounds and tumors. In this review, we discuss the role of MSCs in OS and the potential applications of MSCs in OS treatment. One of the promising clinical applications of MSCs is as a carrier to deliver anti-cancer agents. However, we have to consider the consequence that the recruited MSCs may exhibit their OS-promoting effects. Under this circumstance, it is indispensable for us to evaluate the anti-cancer agents’ OS-inhibiting effects and MSCs’ OS-promoting effects. Another promising application is to target upstream or downstream modulators to block the cross-talk between OS cells and MSCs. Yet, the complexity and multiplicity of the communication networks make it difficult to find an effective antagonist. AMD3100 (inhibiting CXCR4) [49] and 1-MT (inhibiting indoleamine 2,3-dioxygenase) [50] are current frequently used antagonists. Although these antagonists haven’t been used for the treatment of OS, investigations on them are ongoing, and the potential of MSCs may be massive in the future.

## Abbreviations

ASC: Adipose tissue-derived MSC
BM-MSC: Bone marrow MSC
BMP: Bone morphogenetic protein
CSC: Cancer stem cell
IFN: Interferon
IL: Interleukin
MCP: Monocyte chemoattractant protein
MIF: Macrophage inhibition factor
MSC: Mesenchymal stem cell
N-MSC: Normal tissue MSC
OS: Osteosarcoma
PDGF: Platelet derived growth factor
PIGF: Placenta growth factor
SDF: Stromal-derived factor
TAF: Tumor-associated fibroblast
TGF: Transforming growth factor
TME: Tumor microenvironment
T-MSC: Tumor tissue MSC
TNF: Tumor necrosis factor
VEGF: Vascular endothelial growth factor
WJ-MSCs: Wharton’s jelly derived MSC.
